The article "Comparative assessment of various supplementary diets on commercial honey bee (Apis mellifera) health and colony performance" was retracted in 2022. Reasons: compromised peer review; a conflict of interest; concerns about the authorship.

# Comparative assessment of various supplementary diets on commercial honey bee (*Apis mellifera*) health and colony performance

**DOI:** 10.1371/journal.pone.0258430

**Published:** 2021-10-11

**Authors:** Saboor Ahmad, Khalid Ali Khan, Shahmshad Ahmed Khan, Hamed A. Ghramh, Aziz Gul

**Affiliations:** 1 Department of Entomology, Faculty of Crop and Food Sciences, Pir Mehr Ali Shah (PMAS) Arid Agriculture University Rawalpindi, Rawalpindi, Pakistan; 2 Institute of Apicultural Research/Key Laboratory of Pollinating Insect Biology, Ministry of Agriculture, Chinese Academy of Agricultural Sciences, Beijing, China; 3 Research Centre for Advance Material Science (RCAMS), King Khalid University, Abha, Saudi Arabia; 4 Unit of Bee Research and Honey Production, Faculty of Science, King Khalid University, Abha, Saudi Arabia; 5 Biology Department, Faculty of Science, King Khalid University, Abha, Saudi Arabia; 6 Department of Animal Science, Faculty of Agriculture, Hatay Mustafa Kemal University, Hatay, Turkey; Anhui Agricultural University, CHINA

## Abstract

A healthy honey bee stock is critical to the beekeeping industry and the sustainability of the ecosystem. The quality of the supplemental diet influences the development and strength of the colony, especially during the pollen dearth period in the surrounding environment. However, the extent to which pollen substitute protein feeding affects honey bee colony parameters is not fully known. We conducted this study to test the influence of various supplemental diets on foraging effort, pollen load, capped brood area, population density, and honey yield. The treatment groups were supplied with patties of pollen substitute diets, whereas sugar syrup was given to the control group. Our results indicated that honey bees consumed a significantly higher amount of Diet 1 (45 g soybean flour + 15 g Brewer’s yeast + 75 g powdered sugar + 7.5 g skimmed milk + 7.5 g date palm pollen + 200 mL sugar syrup supplement with Vitamin C) followed by others supplemented diets. Further, pollen load, worker-sealed brood area, population strength, and honey yield differed significantly when Diet 1 was consumed instead of other supplemental diets. The proportion of biological parameters was less in the control group as compared to other treatments. This study highlights the potential of supplemental diets to improve the bee’s health and colony development when the pollens availability and diversity are insufficient.

## Introduction

The honey bee is the most important eusocial insect, that plays a critical role in maintaining the natural ecosystem and is directly beneficial to mankind [1]. They produce honey, royal jelly, propolis, and beebread, and provide pollination services for both wild and agricultural crops [1–4]. Although, multiple factors negatively affect bee populations including habitat loss, predators, parasites, diseases, pesticides exposure, and climatic changes [5, 6]. Foraging dynamics of the bees are implicated in the maintenance of populations and their colony heath [7, 8]. Similarly, sufficient food availability in the honey bee colony is necessary for the growth and development.

The article "Comparative assessment of various supplementary diets on commercial honey bee (Apis mellifera) health and colony performance" was retracted in 2022. Reasons: compromised peer review; a conflict of interest; concerns about the authorship.

Honey bees can visit various food sources at the same time and covers the distance of around 10 kilometers to collect primary food resources such as nectar and pollen that are stored in their colonies as honey and beebread [9]. Among these, nectar is the main source of carbohydrates necessary to meet energy requirements [10, 11]. Honey bees obtain macro and micronutrients including proteins, minerals, vitamins, and lipids from pollen that are essential for brood rearing, maturation, adult longevity, and overall colony development [12, 13]. Fatty acids contents and the nutritional components of pollen varies greatly between the diversity of plant species [14], and are directly linked to honey bee health [15]. Notably, the nutritional value of pollen may be more precisely defined by its amino acid components rather than by its total protein contents, because its nutritional value is decreased when there are insufficient amounts of essential amino acids present [16, 17].

Determining the consumption of foods for honey bees is a complex phenomenon; because nutritional requirements are highly variable between different castes and life stages, inter and intraseasonal variability in terms of food availability. Further, supplemental feeding is highly variable during beekeeping practices [18]. During winter or the dry season, when food resources become scarce it affects the queen egg-laying capacity, less worker bees availability, and increases the rates of absconding or abandonment [19]. In the Middle East, higher temperatures and dry conditions in the summer season are the main factors contributing to honey bee mortalities. This is due to the lower blossoming of plants, low availability of pollens caused by heat stress which is the essential food source for forager bees [20]. Thereby, an artificial pollen substitute diet is required to maintain the strong colony health for honey production and pollination [21].

Scientists around the world has formulated various artificial diets recipes for honey bees based on their nutritional requirements of pollen and honey to maintain the better colony health [22, 23]. During a certain period of the year, floral scarcity occurs due to seasonal changes and environmental stressors in various parts of the world [22, 24]. Therefore, it is important to provide pollen substitute to bee colonies for survival and development, which is calculated through various parameters such as reproductive performance, disease resistance, hive weight gain, dietary consumption or by measuring the area of the worker broods [25–28]. A large number of diets formulations have been developed by combining various ingredients including soybean flour, soya flour, parched gram, brewer’s yeast, guar meal, egg yolk powder, pea powder, skimmed milk powder, protein hydrolysate powder, casein, fish meal, and rice bran [29–31]. To my best knowledge, no study thoroughly deals with the impact of supplemental diet on the different parameters of honey bee colonies.

The article "Comparative assessment of various supplementary diets on commercial honey bee (Apis mellifera) health and colony performance" was retracted in 2022. Reasons: compromised peer review; a conflict of interest; concerns about the authorship.

This study was conducted to determine the efficacy of supplemental diets on different parameters of honey bee colonies including diet consumption rate, worker sealed brood area, population density, and honey yield. Further, to investigate the effects of supplemented diets on the foraging effort and pollen collection. This study may develop the guidelines for beekeepers on how to manage and innovatively work in the beekeeping industry to solve the food scarcity problem of honey bees during the pollen shortage times.

## Materials and methods

The study was conducted at Barani Agriculture Research Institute Chakwal, the experiment was conducted on randomly selected colonies. The current study was performed with fifteen honey bee (*Apis mellifera*) colonies from June to October 2020. These colonies were equally divided into five groups of three colonies of each, which were kept in the Langstroth hive. Honey bee colonies with no clinical disease sign were used for this study. For consistency, each colony contained an equal size population, unsealed and sealed worker broods, pollen area, and honey frame. All colonies were managed according to recommended practices followed throughout the experiment.

### Preparation of pollen substitute diet and feeding

These pollen substitute diets contained a suitable amount of proteins, carbohydrates, minerals, and lipids. These products were available at a cheap price in the local market. The following supplemental diets were prepared.

Diet 1 = 150 g (45 g soybean flour + 15 g Brewer’s yeast + 75 g powdered sugar + 7.5 g skimmed milk + 7.5 g date palm pollen + 200 mL sugar syrup supplement with Vitamin C).
Diet 2 = 150 g (60 g soybean flour + 30 g Brewer’s yeast + 60 g powdered sugar + 200 mL sugar syrup).
Diet 3 = 150 g (45 g maize flour + 30 g Brewer’s yeast + 75 g powdered sugar + 200 mL sugar syrup).
Diet 4 = 150 g (60 Germinated pea flour + 30 g Brewer’s yeast + 60 g powdered sugar + 200 mL sugar syrup).
Diet 5 = Control (1 liter of 50% sugar syrup).

The article "Comparative assessment of various supplementary diets on commercial honey bee (Apis mellifera) health and colony performance" was retracted in 2022. Reasons: compromised peer review; a conflict of interest; concerns about the authorship.

The mixture of various supplemental diets and sugar syrup were prepared separately and were mixed thoroughly in a dough maker (Hobart dough mixer, model A200) to make a smooth patty. All supplemental diets were stuffed in patties that were directly placed on brood frames and covered with a plastic sheet to avoid drying. Patties were prepared freshly and each experimental colony received 100 grams of each supplemental diet at 7 days intervals till the end of the experiment. While those honey bee colonies that did not feed on pollen substitute diets were considered as a control. However, the control group received a one-liter sugar solution (1:1 with water) per week to prevent the starvation of bees. The following parameters were measured to check the efficiency of pollen substitutes on colony health.

### Diet consumption

The amount of supplement diet consumption was measured as a difference between the fresh weight of the supplemental diet and the weight of the remaining diet one week after provision to the colony (g per colony) (Patties consumption = beginning patty weight-ending patty weight). The total food consumed by each group was also calculated at the end of the experiment. Pollen traps were mounted at the entrance of each hive to encourage bees to consume the maximum quantity of pollen substitute diets.

### Foraging activity and pollen weight

The foraging activity was measured visually at the hive entrance to count the number of bees return to their respective hive with and without corbicular pollen loads over the 15 minutes between the hours of 9:00 AM, 12:00 PM, and 15:00 PM. The quantity of pollen collected by each colony was estimated by weighing the content of the pollen traps every week.

### Worker sealed brood area

The capped worker brood area was measured after every 12 days with the help of a modified grid system. The grid consisted of squares with an area of one inch^2^ each [32, 33]. The obtained values were converted into cm^2^ by multiplying with 6.45 factors [31]. The grid was placed on the brood frame area, and the comb area occupied by the sealed brood was measured.

### Honey bee population strength

The mean honey bee population was measured by the number of frames covered with bees [34]. The adult honey bee population was estimated after every 12 days by measuring the total number of frames entirely covered by bees. A fully covered frame from each side was considered to be two thousand bees based on earlier assessment.

### Honey production

At the end of the flowering season, the honey yield was estimated by the weight of the comb before and after the honey extraction process [35]. The weight difference of comb is considered as harvestable honey per colony.

The article "Comparative assessment of various supplementary diets on commercial honey bee (Apis mellifera) health and colony performance" was retracted in 2022. Reasons: compromised peer review; a conflict of interest; concerns about the authorship.

### Statistical analysis

The total amount of patty consumed, foraging activity, pollen weight, sealed worker brood area, honey bee population, and honey yield data were compared across the treatments. The results were calculated as (Mean ± Standard Error) by SPSS software (version 26) according to the analysis of variance (ANOVA). The graphs were made using GraphPad Prism software (version 7.03). The significant difference was estimated using Student’s *t*-test between two groups, and one-way ANOVA was used to test a statistically significant difference between more than two groups. Further, the Tukey post-hoc test was performed for multiple comparisons between groups at the 0.05 level.

## Results

### Supplemental diet consumption

There was a statistically significant difference observed between the various supplement diet consumption over the time of observation (F (3,188) = 129.479, P = 0.001). Honey bee consumed a significantly higher amount of Diet 1 (106 ± 2.16 g) in comparison to Diet 3 (73.79 ± 1.73 g) and Diet 4 (68.43 ± 1.38 g), respectively (**Fig 1A**). Hence, there was no significant difference observed between Diet 1 and Diet 2 consumption (**Table 1**). Further, honey bee colonies consumed maximum Diet 1 (131.33 ± 1.86 g) followed by Diet 2 (112.33 ± 6.17 g), Diet 3 (93.67 ± 4.66 g), and Diet 4 (83.33 ± 1.85 g) per week, respectively (**Fig 1B**).

**Fig 1:** Mean weight (g) of supplement diet consumed by honey bee colonies in each treatment. (A), the maximum weight (shows as mean ± standard error) of diet consumption by honeybee colonies over the time of observation. (B), the maximum weight (shows as mean ± standard error) of various diets consumed by honey bee colony per week. The different small letter within each data represents statistically significant differences (p<0.05).

**Table 1:** Effect of various supplemental diets on honeybee health and colony performance.

Treatment	Diet consumption (g/colony)	Pollen weight (g/colony)	Worker sealed brood area (cm2)	Honey bee population (frames/colony)	Honey yield (kg/colony)
	Mean ± S. Error	Mean ± S. Error	Mean ± S. Error	Mean ± S. Error	Mean ± S. Error
Diet 1	106.08 ± 2.15 a	77.94 ± 0.94 a	2277.29 ± 28.67 a	14.54 ± 0.21 a	13.00 ± 1.15 a
Diet 2	101.86 ± 1.34 a	60.02 ± 1.00 b	1883.79 ± 13.41 b	11.95 ± 0.16 b	9.67 ± 0.88 b
Diet 3	73.79 ±1.73 b	54.85 ±1.63 c	1747.58 ± 7.11 c	10.92 ± 0.17 c	7.67 ± 1.45 c
Diet 4	68.44 ± 1.38 b	38.79 ± 0.98 d	1452 ± 18.17 d	8.58 ± 0.18 d	5.33 ± 0.33 d
Diet 5	_	25.48 ± 0.79 e	843.96 ± 10.79 e	6.5 ± 0.19 e	3.33 ± 0.67 e

The different small letter within each column represents statistically significant differences (p<0.05).

The article "Comparative assessment of various supplementary diets on commercial honey bee (Apis mellifera) health and colony performance" was retracted in 2022. Reasons: compromised peer review; a conflict of interest; concerns about the authorship.

### Foraging effort and pollen load

Foraging effort was recorded by the number of bees returned to their respective colony with corbicular pollen (**Fig 2A and 2B**). Multiple comparisons confirmed that foraging effort differed significantly between the diets at 9:00 AM as an observation period (F (4,75) = 31.830, P = 0.001). Similarly, a significant difference between the diets at “12:00 PM” (F (4,75) = 40.554, P = 0.001) and at “15:00 PM” (F (4,75) = 41.515, P = 0.001) were found (**Fig 2A**). The maximum number of honey bees with pollen were observed in the case of Diet 1 (76.33 ± 3.92), and a smaller number of bees were observed in control (33.33 ± 1.67) per week (**Fig 2B**).

**Fig 2:** The foraging effort and pollen collection weight (shows as mean ± standard error) by consumption of various diets. (A), the mean number of bees with pollen was recorded at 9:00 AM, 12:00 PM, and 15:00 PM. (B), the mean number of foragers were detected per week per colony. (C), the mean collected pollen weight by use of various diets. (D), the mean collection of pollen weight per week per colony. The different small letter within each data represents statistically significant differences (p<0.05).

The mean collection of pollen weight differed significantly between the diets over the time of inspection (F (4,235) = 330.178, P = 0.001). The highest pollen weight (77.94 ± 0.94 g) was detected by the use of Diet 1 in comparison to other diets, whereas the less pollen weight (25.48 ± 0.80 g) in control (**Fig 2C**). Similarly, the maximum pollen weight was recorded by the consumption of Diet 1 (88.67 ± 5.55 g/colony) and less weight of pollen per colony was detected in control (19.00 ± 0.58 g) per week (**Fig 2D**).

### Worker sealed brood area

The worker-sealed brood area differed significantly between the consumption of various diets (F (4,115) = 955.214, P = 0.001). The maximum sealed brood area was observed in the consumption of Diet 1 (2277. 29 ± 28.68 cm^2^), whereas less brood area was detected in control (843.95 ± 10.79 cm^2^) over the time of observation (**Fig 3A**). The sealed brood area was significantly higher after the consumption of Diet 1 (2333.33 cm^2^) followed by other diets, and less sealed brood was found in control (749.67 cm^2^) over the twelve days intervals (**Fig 3B**).

**Fig 3:** The worker sealed brood area (shows as mean ± standard error) recorded after the consumption of various diets. (A), the mean sealed brood area over the time of observation. (B), the mean sealed brood area after each twelve days intervals. The different small letter within each data represents statistically significant differences (p<0.05).

The article "Comparative assessment of various supplementary diets on commercial honey bee (Apis mellifera) health and colony performance" was retracted in 2022. Reasons: compromised peer review; a conflict of interest; concerns about the authorship.

### Honey bee population density

The impact of various supplemental diets on comb covered with bees were described in (**Fig 4**). The number of frames covered with bees differed significantly by consuming various diets (F (4,115) = 285.507, P = 0.001). The mean number of frames covered with bees were significantly higher in the case of Diet 1 (14.55 ± 0.21) compared to other diets, whereas the number of bee frames were (6.5 ± 0.19) smaller in control groups (**Fig 4A**). The maximum number of bee frames were recorded after the consumption of Diet 1 (15.67 ± 0.33), whereas the lower number of frames with bees were found in control (5.67 ± 0.33) over the twelve days intervals (**Fig 4B**).

**Fig 4:** The number of frames (shows as mean ± standard error) with bees recorded after the consumption of various diets. (A), the mean number of frames over the time of observation. (B), the mean number of frames with bees after each twelve days intervals.

### Honey yield

The amount of honey yield per colony after the consumption of various diet was analysed (**Fig 5**). Honey yield differed significantly after the use of various diets among honey bee colonies (F (4,10) = 14.804, P = 0.001).

**Fig 5:** The amount of honey yield (shows as mean ± standard error) per colony was recorded after the consumption of various diets. The different small letter within each data represents statistically significant differences (p<0.05).

The highest honey yield per colony was found in Diet 1 (13.00 ± 1.15 kg/colony) and Diet 2 (9.67 ± 0.88 kg/colony), and low yield was detected in control that was 3.33 ± 0.67 kg colony^-1^ (**Table 1**).

## Discussion

In this study, we compared the effect of various supplementary diets on honey bee health and colony development. Our result revealed that supplement diets have a significant impact on foraging effort and pollen collection (**Table 1**). The mean weight of bee collected pollen trapped at the colony entrance was considered a direct assessment of foraging success. The annual availability of pollen for bee colonies varies according to variation in floral sources and population density of bee colonies. The adequate flora of honey bee interest is not available throughout the year, so the provision of artificial pollen supplements and pollen substitutes have been used to maintain the strength of bee colony by increasing brood area and longevity of bees [36]. While these supplemental diets and pollen substitutes may represent a temporary solution to prevent bee losses in unfavorable foraging situations but it cannot possibly be sustained as a long-term solution in a pollen dearth period.

The article "Comparative assessment of various supplementary diets on commercial honey bee (Apis mellifera) health and colony performance" was retracted in 2022. Reasons: compromised peer review; a conflict of interest; concerns about the authorship.

Further, the consumption of a supplemental diet increased the worker-sealed brood area, honey bee population density, and honey yield compared to control groups (**Table 1**). Sihag and Gupta [37], Lamontagne-Drolet, Samson-Robert [38], and Islam, Mahmood [39] reported a similar result that the surface of sealed brood area was increased after the consumption of various supplements and pollen substitutes by honey bees. Similarly, Abd El-Wahab, Ghania [31] represented the same results that sealed brood area increased in supplementarily fed bee colonies in relation to un-fed bee colonies. DeGrandi-Hoffman, Wardell [34, 39, 40] revealed that supplemental diets increased the population density in comparison to the non-supplemented control group. Honey yield also increased significantly in those bee colonies which fed on supplemental diets than the control colonies that fed only sugar syrup [26, 31, 39]. All supplemental diets tests here were not equally effective in stimulating the various biological activities of honey bee colonies. However, Huang [41] and Amro, Omar [42] documented that honey bee usually prefers natural pollen as compared to pollen substitute diets.

Generally, supplemental diets led to a higher amount of protein contents in the bee in comparison to control bee colonies, regardless of the existence of bee pollen trap. Expectedly, bee colonies with the absence of pollen traps contain a higher amount of protein content as they were able to use both natural pollen and supplemental diets. However, supplemented bee colonies which were restricted to consume natural pollen also had more protein content as compared to control.

Our inferences regarding supplemental diet consumption are limited because most of the bee colonies used various amount of diet quantity per week. Therefore, we cannot determine the exact amount of supplemental diet consumed by each bee colony on a daily basis. We also do not know how bees use different supplemental protein diets.

Additionally, more field studies are needed to determine the effect of these supplemental diets on honey bee health and colony performance. This study may help the beekeepers to design more appropriate food materials, that minimize waste and increase the nutritional intake of their bee colonies.

## Conclusions

We concluded that supplemental diets have a great impact on honey bee health and colony developmental parameters. Honey bee colonies have a significantly higher amount of pollen load, worker-sealed brood area, population density, and honey yield after the consumption of diet supplements than the control group. However, Diet 1 (45 g soybean flour + 15 g Brewer’s yeast + 75 g powdered sugar + 7.5 g skimmed milk + 7.5 g date palm pollen + 200 mL sugar syrup supplement with Vitamin C) had a significant impact on honey bee colony developmental parameters followed by Diet 2, Diet 3, Diet 4, and control, respectively. The present study highlights the importance of supplemental diets for the honey bee colonies when the pollens are not available in sufficient amount. Further studies are needed to investigate the effect of these supplements on various physiological parameters of honey bee races during different environmental conditions.

The article "Comparative assessment of various supplementary diets on commercial honey bee (Apis mellifera) health and colony performance" was retracted in 2022. Reasons: compromised peer review; a conflict of interest; concerns about the authorship.

## References

[1] KleinA-M, VaissiereBE, CaneJH, Steffan-DewenterI, CunninghamSA, KremenC, et al. Importance of pollinators in changing landscapes for world crops. Proc Royal Soc B 2007;274(1608):303–13. doi: 10.1098/rspb.2006.3721 17164193PMC1702377

[2] RequierF, GarneryL, KohlPL, NjovuHK, PirkCW, CreweRM, et al. The conservation of native honey bees is crucial. Trends Ecol Evol. 2019;34(9):789–98. doi: 10.1016/j.tree.2019.04.008 31072605

[3] AhmadS, KhalofahA, KhanSA, KhanKA, JilaniMJ, HussainT, et al. Effects of native pollinator communities on the physiological and chemical parameters of loquat tree (Eriobotrya japonica) under open field condition. Saudi J Biol Sci. 2021;28(6):3235–41. doi: 10.1016/j.sjbs.2021.02.062 34121860PMC8176055

[4] AnjumSI, UllahA, KhanKA, AttaullahM, KhanH, AliH, et al. Composition and functional properties of propolis (bee glue): A review. Saudi J Biol Sci. 2019;26(7):1695–703. doi: 10.1016/j.sjbs.2018.08.013 31762646PMC6864204

[5] SmithKM, LohEH, RostalMK, Zambrana-TorrelioCM, MendiolaL, DaszakP. Pathogens, pests, and economics: drivers of honey bee colony declines and losses. EcoHealth. 2013;10(4):434–45. doi: 10.1007/s10393-013-0870-2 24496582

[6] GoulsonD, NichollsE, BotíasC, RotherayEL. Bee declines driven by combined stress from parasites, pesticides, and lack of flowers. Science. 2015;347(6229).10.1126/science.125595725721506

[7] VaudoAD, TookerJF, GrozingerCM, PatchHM. Bee nutrition and floral resource restoration. Curr Opin Insect Sci. 2015;10:133–41. doi: 10.1016/j.cois.2015.05.008 29588000

[8] KhanKA, GhramhHA. Pollen source preferences and pollination efficacy of honey bee, Apis mellifera (Apidae: Hymenoptera) on Brassica napus crop. J King Saud Univ Sci. 2021:101487.

[9] WrightGA, NicolsonSW, ShafirS. Nutritional physiology and ecology of honey bees. Annu Rev Entomol. 2018;63:327–44. doi: 10.1146/annurev-ento-020117-043423 29029590

[10] Abou-ShaaraH. The foraging behaviour of honey bees, Apis mellifera: a review. Vet Med (Praha). 2014;59(1).

[11] KhanKA, GhramhHA, AhmadZ, El-NiweiriMA, MohammedMEA. Honey bee (Apis mellifera) preference towards micronutrients and their impact on bee colonies. Saudi J Biol Sci. 2021;28(6):3362–6. doi: 10.1016/j.sjbs.2021.02.084 34121873PMC8175997

The article "Comparative assessment of various supplementary diets on commercial honey bee (Apis mellifera) health and colony performance" was retracted in 2022. Reasons: compromised peer review; a conflict of interest; concerns about the authorship.

[12] LoidlA, CrailsheimKJJoCPB. Free fatty acids digested from pollen and triolein in the honeybee (Apis mellifera carnica Pollmann) midgut. J Comp Physiol B. 2001;171(4):313–9. doi: 10.1007/s003600100178 11409628

[13] ArienY, DagA, ShafirS. Omega-6: 3 ratio more than absolute lipid level in diet affects associative learning in honey bees. Front Psychol. 2018;9:1001. doi: 10.3389/fpsyg.2018.01001 29971031PMC6018467

[14] T’aiHR, CaneJH. Pollen nutritional content and digestibility for animals. Pollen pollination 2000:187–209.

[15] AlauxC, DuclozF, CrauserD, Le ConteY. Diet effects on honeybee immunocompetence. Biol Lett. 2010;6(4):562–5. doi: 10.1098/rsbl.2009.0986 20089536PMC2936196

[16] CookSM, AwmackCS, MurrayDA, WilliamsIH. Are honey bees’ foraging preferences affected by pollen amino acid composition? Ecol Entomol. 2003;28(5):622–7.

[17] Al-KahtaniSN, TahaE-K, KhanKA, AnsariMJ, FaragSA, ShawerDM, et al. Effect of harvest season on the nutritional value of bee pollen protein. PLoS One. 2020;15(12):e0241393. doi: 10.1371/journal.pone.0241393 33370277PMC7769433

[18] RodneyS, PurdyJ. Dietary requirements of individual nectar foragers, and colony-level pollen and nectar consumption: a review to support pesticide exposure assessment for honey bees. Apidologie. 2020;51(2):163–79.

[19] MoraisMM, TurcattoAP, FrancoyTM, GonçalvesLS, CappelariFA, De JongD. Evaluation of inexpensive pollen substitute diets through quantification of haemolymph proteins. J Apic Res. 2013;52(3):119–21.

[20] AwadAM, OwayssAA, AlqarniAS. Performance of two honey bee subspecies during harsh weather and Acacia gerrardii nectar-rich flow. Scientia Agricola. 2017;74(6):474–80.

[21] Di PasqualeG, SalignonM, Le ConteY, BelzuncesLP, DecourtyeA, KretzschmarA, et al. Influence of pollen nutrition on honey bee health: do pollen quality and diversity matter? PLoS One. 2013;8(8):e72016. doi: 10.1371/journal.pone.0072016 23940803PMC3733843

[22] ParayBA, KumariI, HajamYA, SharmaB, KumarR, AlbeshrMF, et al. Honeybee nutrition and pollen substitutes: A review. Saudi J Biol Sci. 2021;28(1):1167. doi: 10.1016/j.sjbs.2020.11.053 33424413PMC7783834

[23] Paiva JPLMPaiva HM, Esposito EMorais MM. On the effects of artificial feeding on bee colony dynamics: a mathematical model. PLoS One. 2016;11(11):e0167054. doi: 10.1371/journal.pone.0167054 27875589PMC5119823

[24] Feliciano-CardonaS, DökeMA, AlemanJ, Agosto-RiveraJL, GrozingerCM, GirayT. Honey bees in the tropics show winter bee-like longevity in response to seasonal dearth and brood reduction. Front Ecol Evol. 2020;8:336.

The article "Comparative assessment of various supplementary diets on commercial honey bee (Apis mellifera) health and colony performance" was retracted in 2022. Reasons: compromised peer review; a conflict of interest; concerns about the authorship.

[25] KumarR, MishraR, AgrawalO. A Study on Consumption of some artificial diet formulations by Apis mellifera colonies maintained at Panchkula & Gwalior. J Entomol Res. 2013;37(2):123–7.

[26] ShehataI. Evaluation of Carniolan and Italian honey bee colonies fed on artificial diets in dearth and flowering periods under Nasr city conditions. Int J Environ. 2016;5(2):19–25.

[27] GemedaTK. Testing the effect of dearth period supplementary feeding of honeybee (Apis mellifera) on brood development and honey production. Int J Adv. 2014;2(11):319–24.

[28] DeGrandi-HoffmanG, ChenY, RiveraR, CarrollM, ChambersM, HidalgoG, et al. Honey bee colonies provided with natural forage have lower pathogen loads and higher overwinter survival than those fed protein supplements. Apidologie. 2016;47(2):186–96.

[29] Winston MPC L. Effects of two pollen substitutes on brood mortality and length of adult life in the honey bee. J Apic Res. 1983;22:49–52.

[30] KumariI, KumarR. Pollen Substitute Diet for Apis Mellifera: Consumption and Effects on Colony Parameters in Sub-Tropical Himalaya. Indian J Agric Res. 2020;54(2).

[31] Abd El-WahabT, GhaniaA, ZidanE. Assessment a new pollen supplement diet for honey bee colonies and their effects on some biological activities. Int J Agric. 2016;12(1):55–62.

[32] AmirO, PevelingR. Effect of triflumuron on brood development and colony survival of free‐flying honeybee, Apis mellifera L. J Appl Entomol. 2004;128(4):242–9.

[33] MattilaHR, OtisGW. Dwindling pollen resources trigger the transition to broodless populations of long‐lived honeybees each autumn. Ecol Entomol. 2007;32(5):496–505.

[34] DeGrandi-HoffmanG, WardellG, Ahumada-SeguraF, RindererT, DankaR, PettisJ. Comparisons of pollen substitute diets for honey bees: consumption rates by colonies and effects on brood and adult populations. J Apic Res. 2008;47(4):265–70.

[35] MahmoodR, WagchoureES, SarwarG. Influence of supplemental diets on Apis mellifera L. colonies for honey production. Pak J Agric Res. 2013;26(4).

[36] SafariA, KevanPG, AtkinsonJL. Feed-Bee: A new bee feed is added to the menu. Bee Culture. 2006;134(1):47–8.

[37] SihagRC, GuptaM. Development of an artificial pollen substitute/supplement diet to help tide the colonies of honeybee (Apis mellifera L.) over the dearth season. J Apic Sci. 2011;55(2).

[38] Lamontagne-DroletM, Samson-RobertO, GiovenazzoP, FournierV. The impacts of two protein supplements on commercial honey bee (Apis mellifera L.) colonies. J Apic Res. 2019;58(5):800–13.

[39] IslamN, MahmoodR, SarwarG, AhmadS, AbidS. Development of pollen substitute diets for Apis mellifera ligustica colonies and their impact on brood development and honey production. Pak J Agric Res. 2020;33(2):381–8.

The article "Comparative assessment of various supplementary diets on commercial honey bee (Apis mellifera) health and colony performance" was retracted in 2022. Reasons: compromised peer review; a conflict of interest; concerns about the authorship.

[40] SihagRC, GuptaM. Testing the Effects of Some Pollen Substitute Diets on Colony Build up and Economics of Beekeeping vvith Apis mellifera L. J Entomol. 2013;10(3):120–35.

[41] HuangZ. Pollen nutrition affects honey bee stress resistance. Terr Arthropod Rev. 2012;5(2):175–89.

[42] AmroA, OmarM, Al-GhamdiA. Influence of different proteinaceous diets on consumption, brood rearing, and honey bee quality parameters under isolation conditions. Turkish J Vet Anim Sci. 2016;40(4):468–75.

